# Maffucci syndrome and soft tissue sarcoma: a case report

**DOI:** 10.1186/1477-7800-6-2

**Published:** 2009-01-13

**Authors:** Fernando César Toniazzi Lissa, Juliana Sonego Argente, Geórgia Nunes Antunes, Franciani de Oliveira Basso, Janara Furtado

**Affiliations:** 1 Department of Surgical Oncology, Hospital São José, Criciúma, Brazil; 2 Department of Internal Medicine, Hospital São José, Criciúma, Brazil

## Abstract

**Background:**

Maffucci syndrome, a congenital mesodermal dysplasia characterized by multiple enchondromas and hemangiomas, was first described in 1881, and 200 cases have been reported in the literature since then. Its etiology is unknown, there is no predilection for race or sex, and the development of lesions usually occurs in puberty. The risk of sarcomatous transformation is about 25%.

**Case presentation:**

The initial investigation of the case reported here focused on the diagnosis and treatment of malignancy, and the first diagnostic hypothesis was thrombosed hemangioma. After histopathologic confirmation of soft tissue sarcoma, examinations were performed to stage the tumor and enchondromas were found in ribs. The final diagnosis was Maffucci syndrome with malignant transformation.

**Conclusion:**

Treatment should aim at symptom relief and early detection of malignancies; no therapy is indicated for asymptomatic patients. As in the case reported here, bone or soft tissue lesions that grow or become painful should be biopsied.

## Background

Maffucci syndrome was first described in 1881, but its etiology remains unknown. About 200 cases have been described in the literature to date [1,2]. This syndrome is characterized by multiple enchondromas, hemangiomas and, less often, lymphangiomas [1-3]. Enchondromas are benign cartilaginous tumors that may develop in any site, are most frequently found in phalanges and long bones, but may also affect the tibia, fibula, humerus, ribs or cranium. Soft tissue tumors usually develop with the bone lesions [1,3].

This congenital mesodermal hyperplasia is nonhereditary, and patients are usually asymptomatic at birth. Symptoms usually develop in puberty [2].

The risk of malignant change is about 25%. Sarcomatous transformation may be seen in bones and soft tissue lesions, but is more frequently found in enchondromas, and its incidence ranges from 15 to 57% [1].

This report describes the case of a 29-year-old patient with a diagnosis of Maffucci syndrome with malignant transformation and a tumor in the right thigh diagnosed as retiform hemangioendothelioma.

## Case presentation

A 29-year-old white woman presented with a tumor that had appeared on the right thigh two years before. Physical examination revealed a hard nodule about five centimeters in diameter with no signs of inflammation. Ultrasound showed a heterogeneous tumor measuring 5.0 × 6.5 × 4.5 cm and coarse calcifications within the tumor. Because of hemangiomas in upper extremities, the initial hypothesis was thrombosed hemangioma.

Histopathological analysis of excisional biopsy specimen showed fusiform and vasoformative tissue. Immunohistochemical analysis suggested a well-differentiated myxoid liposarcoma.

After the diagnosis of soft tissue sarcoma, complete tumor staging was performed using chest radiographs and CT, which showed lytic bone lesions in fourth and seventh anterior ribs, and nuclear MRI of right thigh, which showed a large, predominantly cystic and heterogeneous lesion. Therefore, radical tumor resection was performed. Material was sent to the Mayo Clinic, and the final diagnosis was a low-grade vascular neoplasm consistent with retiform hemangioendothelioma and not liposarcoma, as previously thought.

After one-year follow-up, the patient noticed a new tumor on the right thigh and inguinal region, and biopsy confirmed lymph node metastasis. Chest CT revealed several lung lesions, but etiology was not confirmed by biopsy. Chemotherapy with doxorubicin was initiated, and full clinical response was achieved.

## Conclusion

Maffucci syndrome is a rare clinical entity characterized by multiple enchondromas, hemangiomas and, less often, lymphangiomas [1-3]. The disease often develops in puberty (78%), but symptoms are present at birth or are observed in the first year of life in 25% of the cases [2]. In the case described here, the patient reported that symptoms were first noticed at the end of the second decade of life, an unusual age, but already reported in other cases.

Bone changes are caused by congenital defects in endochondral ossification and lead to deficits in final bone growth and bone irregularities. Enchondromas are more often found in hand phalanges, metacarpal bones, foot bones, tibia, fibula, radius and ulna [1,3]. Distribution is asymmetric, and bone lesions may range from painless edema to pathological fractures. Other bones may be affected, although not as often, as in the case described here, in which ribs were primarily affected [1]

Hemangiomas are usually found along soft tissues as bluish nodules, but may also be found in internal organs and mucous membranes, particularly in the brain, eyes, and gastrointestinal tract [1].

Pathological fractures are found in 26% of the cases; other possible complications are hemorrhage, short stature, pleural effusion and cranial nerve paralysis due to endochondral compression [1].

The differential diagnosis from Ollier disease should be established because, although chondrodysplasia is found in both, Maffucci syndrome is associated with risk of malignancy [2]. Sarcomatous transformation occurs in 25% of the cases, mainly in enchondromas, and may also occur in soft tissues and bones [1]. The case reported here showed malignant change to retiform hemangioendothelioma, a rare form of soft tissue sarcoma.

Retiform hemangiomas (RHE) are extremely rare low-grade variations of well-differentiated angiosarcoma, characterized by high recurrence rates and low metastatic potential [4]. In the case described here, the patient had lymph node metastasis in addition to a rare sarcoma. The treatment of choice in such case is surgical excision with tumor-free margins [5].

Treatment should aim at symptom relief and early detection of malignancies. Surgical procedures consist of osteotomy and curettage of bone lesion. Other therapeutic options are sclerotherapy, irradiation and vascular lesion surgery. Excision is the procedure of choice for soft tissue tumors [2].

Bone and soft tissue lesions that grow or become painful without a history of trauma should be examined for malignancy and biopsied. No treatment is indicated for asymptomatic patients without malignant transformation, and prognosis is usually good [6].

## Competing interests

The authors declare that they have no competing interests.

## Authors' contributions

FTL carried out overall design of the manuscript and was responsible for the writing of the report. JSA participated in manuscript design and helped to draft the manuscript. GNA was responsible for all the literature review and contributed to the discussion. FOB contributed to case description and gave final approval of the version to be published.

JF conceived the theory behind the report and helped to draft the manuscript. All authors read and approved the final manuscript.

## Consent

Written consent was obtained from the patient or their relative for publication of study.

## References

[B1] Biber C, Ergun P, Turay UY, Erdogan Y, Hizel SB (2004). A case of Maffucci's Syndrome with pleural effusion: ten-year follow-up. Ann Acad Med Singapore.

[B2] Flach HZ, Ginai AZ, Oosterhuis FW (2001). Maffucci Syndrome: radiologic and pathologic findings. Radiographics.

[B3] Jermann M, Eid K, Pfammatter T, Stahel R (2001). Maffucci's Syndrome. Circulation.

[B4] Duke D, Dvorak A, Harris TJ, Cohen LM (1996). Multiple retiform hemangioendothelioma: A low grade angiosarcoma. Am J Dermatopathol.

[B5] Despina I, Panaylotides J, Krasagakis K, Stefanidou M, Manios A, Tosca A (2006). Retiform hemangioendothelioma presenting as bruise-like plaque in an adult woman. Int J Dermatol.

[B6] Lewis RJ, Ketcham AS (1973). Maffucci's Syndrome: Functional and neoplastic sigficance – case report and review of the literature. J Bone Joint Surg Am.

